# Denatured Mammalian Protein Mixtures Exhibit Unusually High Solubility in Nucleic Acid-Free Pure Water

**DOI:** 10.1371/journal.pone.0113295

**Published:** 2014-11-18

**Authors:** Junichiro Futami, Haruna Fujiyama, Rie Kinoshita, Hidenori Nonomura, Tomoko Honjo, Hiroko Tada, Hirokazu Matsushita, Yoshito Abe, Kazuhiro Kakimi

**Affiliations:** 1 Department of Biotechnology, Graduate School of Natural Science and Technology, Okayama University, Okayama, Japan; 2 Department of Immunotherapeutics, The University of Tokyo Hospital, Tokyo, Japan; 3 Department of Protein Structure, Function and Design, Graduate School of Pharmaceutical Sciences, Kyushu University, Fukuoka, Japan; Kermanshah University of Medical Sciences, Islamic Republic of Iran

## Abstract

Preventing protein aggregation is a major goal of biotechnology. Since protein aggregates are mainly comprised of unfolded proteins, protecting against denaturation is likely to assist solubility in an aqueous medium. Contrary to this concept, we found denatured total cellular protein mixture from mammalian cell kept high solubility in pure water when the mixture was nucleic acids free. The lysates were prepared from total cellular protein pellet extracted by using guanidinium thiocyanate-phenol-chloroform mixture of TRIzol, denatured and reduced total protein mixtures remained soluble after extensive dialysis against pure water. The total cell protein lysates contained fully disordered proteins that readily formed large aggregates upon contact with nucleic acids or salts. These findings suggested that the highly flexible mixtures of disordered proteins, which have fully ionized side chains, are protected against aggregation. Interestingly, this unusual solubility is characteristic of protein mixtures from higher eukaryotes, whereas most prokaryotic protein mixtures were aggregated under identical conditions. This unusual solubility of unfolded protein mixtures could have implications for the study of intrinsically disordered proteins in a variety of cells.

## Introduction

Proteins perform an extraordinary array of functions in cells [1]. To understand the behavior of proteins in living cells, we must consider the extremely high intracellular concentrations of macromolecules. The cytoplasmic protein concentration has been estimated to be 100 mg/mL [2], and the total macromolecular concentration (including proteins, lipids, nucleic acids, and sugars) could be as high as 400 mg/mL [3]. Proteins have therefore evolved to exert their biological functions under highly crowded conditions, which raises the question of how they maintain solubility in such a dense milieu. Intrinsically unstructured proteins display unusually high solubility, and studying these molecules may elucidate the mechanisms underlying this phenomenon.

Proteins must fold into unique three-dimensional structures and interact specifically with particular molecules to function correctly. However, some proteins exist in an intrinsically unstructured form, lacking stable secondary and tertiary structural elements, but retaining full functionality. These intrinsically disordered proteins (IDPs) are unfolded *in vitro*, but may adopt functional conformations *in vivo*, although several lines of indirect evidence indicate that IDPs remain disordered in the cell [4], [5]. The capacity for folding or remaining intrinsically unstructured mainly depends on the interplay between water molecules and the characteristic amino acid composition that dictate the hydrophobicity, charge, and flexibility [6], [7]. Generally, IDPs lack bulky hydrophobic residues such as Ile, Leu, and Val, as well as aromatic residues such as Trp, Tyr, and Phe but are enriched in polar residues such as Arg, Gly, Gln, Ser, Pro, Glu and Lys, and the secondary structure-breaking amino acids Gly and Pro [6], [7]. This composition results in high solubility in water despite being highly unstructured. Much work has been done on prediction of IDPs from protein sequences, and this class of proteins are much more abundant in eukaryotes than in prokaryotes [8], [9]. Although the predicted disorder depends on the program used, intrinsically disordered regions (IDRs) account for 8–10% of protein sequences in prokaryotes and 30–41% in eukaryotes [10], [11]. The majority of cellular proteins are predicted to adopt fully folded biologically active conformations, but IDRs are abundant. Unlike globular proteins, IDPs show unusually high solubility following heat treatment. Kim *et al* (2000) demonstrated that 20% of total proteins in Jurkat T-cell lysates are heat-resistant and remain soluble after boiling [12]. The resultant soluble protein fractions are enriched in IDPs and are a valuable resource for proteomic research [13], [14].

It is widely accepted that denaturing proteins exposes hydrophobic residues that are normally buried in the native conformation, and aggregation is mainly mediated by the resulting hydrophobic or electrostatic interactions between individual molecules. Hydrophobic interactions mainly occur between neighboring denatured protein molecules, whereas electrostatic interactions mainly occur between denatured proteins and anionic nucleic acid polymers. Removal of nucleic acids is therefore critical for efficient oxidative refolding of globular proteins from bacterial inclusion bodies [15]. The refolding efficiency can be improved by altering the ionic strength, pH, and using additives [16], but the final yield of refolded protein is often decreased substantially due to the presence of misfolded protein molecules that seed aggregation during purification steps. Poor protein solubility is a commonly encountered problem, and maintaining proteins in soluble conditions is the conventional approach for ensuring biological activity is maintained. The opposite approach of intentional denaturation is unusual, but may work well for maintaining the solubility of IDPs.

The unusual high solubility of mammalian IDPs appeared to be characteristic of proteins from higher eukaryotes, since most prokaryotic protein mixtures aggregated under similar denaturing conditions. Although the detailed mechanism is unclear, this unusual solubility presumably reflects the amino acid composition of eukaryotic IDPs, and likely reflects key evolutionary differences.

## Materials and Methods

### Cell culture

Human cell lines HeLa S3 and HEK293 PEAKrapid, and the mouse cell line B16 melanoma-F10 were purchased from ATCC. All cell lines were cultured in Dulbecco’s modified Eagle’s medium (DMEM) supplemented with 10% fetal bovine serum (FBS, PAA laboratories, Austria) and penicillin/streptomycin (Wako, Osaka, Japan). *S. cerevisiae*, S288C (National Bio-Resource Project of the MEXT, Japan) was grown in YPD media at 30°C for 24 h. *S. aureus* (FDA 209P) in brain Bacto heart infusion medium (BD Biosciences), and *E. coli* BL21 (DE3) (Novagen) in LB medium were grown at 37°C for 24 h. *E. coli* BL21 (DE3) containing pET23a-human β-actin plasmid DNA were used to express human β-actin. Transformed cells were cultured in LB at 37°C, expression was induced with 0.4 mM IPTG, and growth continued for 3 h.

### Isolation of nucleic acid-free total cell proteins

Total cell proteins were isolated using TRIzol (Invitrogen) according to the manufacturer’s instructions. Briefly, sub-confluent mammalian cells cultured on a 100 mm dish were washed twice with PBS, lysed in 5 mL TRIzol, scraped off and transferred to a centrifuge tube. Proteins were recovered in the organic phase following addition of chloroform, and precipitated by addition of 2-propanol. Protein precipitates were extensively washed with 0.3 M GdnHCl in 95% ethanol at least five times, to give a white protein pellet that was washed three times with ethanol. Ethanol-wet pellets were used directly as they were poorly soluble in 6 M GdnHCl after drying. Cell pellets of *S. cerevisiae*, *S. aureus*, *and E. coli* (0.2 g wet weight were dissolved in 1 mL TRIzol and treated as described above.

### Preparation of protein lysates in salt-free water

Total cell proteins were dissolved in 6 M GdnHCl containing 0.1 M Tris-HCl pH 8.5, and the protein concentration was adjusted for each experiment using values determined from the absorbance at 280 nm, assuming 1 absorbance unit at 280 = 1 mg/mL. Disulfide bonds were then reduced with 0.1 M DTT at 37°C for 1 h, and a 0.1 volume of acetic acid was added. The resultant protein solutions were dialyzed extensively against Milli-Q water using a Slide-A-Lyzer (3.5K MWCO, Thermo Fisher Scientific, Waltham, MA) at 4°C for 48 h. The Milli-Q water was changed every few hours initially then every 12–16 h. Residual nucleic acids in TRIzol lysate were determined with Quant-iT PicoGreen dsDNA and RiboGreen RNA Assay Kit (Life Technologies, Carlsbad, CA). To determine the solubility in TRIzol lysates, initial protein concentrations were adjusted to 1 mg/mL before starting dialysis. Aggregated proteins and the remaining soluble proteins were separated by centrifugation at 14,000×*g* for 15 min at 4°C, and each was solubilized in 8 M urea prior to protein concentration measurement using the Bradford protein assay (Bio-Rad Laboratories, Hercules, CA) with bovine serum albumin as a standard.

### Determination of protein solubility in lysates containing additives

Nucleic acid-free total cell protein lysates (TRIzol lysates) from HeLa cells in Milli-Q water and with a protein concentration of 2–3 mg/mL and a pH of 5 and an electrical conductivity <20 µS/cm were used for assays. dNTPs (Thermo) 16S-rRNA and 23S-rRNA from *E. coli* MRE600 (Boehringer Mannheim, Germany), tRNA from baker’s yeast (Type X-SA, Sigma, St. Louis, MO), or DNA from calf thymus (phenol-chloroform extracted, <2000 bp, WAKO) were mixed with TRIzol lysates to give a protein concentration of 0.1 mg/mL, and incubated for 60 min at 4°C. After centrifugation at 14,000×*g* for 15 min at 4°C, the concentration of soluble proteins was determined by Bradford protein assay (Bio-Rad).

### Plasmid transfection and functional assays

Plasmids for expression of the enhanced GFP (pEGFP-N1; Clontech, Mountainview, CA) and firefly luciferase (Luc; pGL3-basic; Promega, Madison, WI) were used to transfect HEK293 PEAKrapid cells using 293 fectin (Invitrogen) which were subsequently cultured for 24 h. To prepare native protein lysates, cells were lysed with Glo Reporter Lysis Buffer (GLB, Promega). The fluorescence intensity of EGFP-containing lysates was analyzed using a Multi Microplate Reader MTP-800 (Hitachi, Japan) at Ex/Em: 480/530 nm. Luminescence of Luc-containing lysates was measured using a steady Glo assay kit (Promega) and Luminometer Junior LB9509 (Berthold Technologies, Dak Ridge, TN).

### Western blotting

Endogenous and transiently expressed reporter protein levels were verified by Western blotting using conventional procedures using the following primary antibodies; anti-β-actin (13E5, Cell Signaling Technologies, Beverly, MA), β-tubulin (Cell Signaling Technologies), GFP (mFX75, Wako), Luciferase (MBL, Nagoya, Japan). Membranes were treated with horseradish peroxidase-conjugated anti-mouse IgG or anti-rabbit IgG (Cell Signaling Technology), and positive signals were measured using a chemiluminescence system.

### NMR

NMR spectra were recorded at 37°C on a Varian Unity INOVA 600 spectrometer (Varian, CA). 3Hmutwil and *S*-carboxymethylated mouse lysozyme were prepared as described previously [17]–[19], and 0.1 mM samples of ^15^N-labeled proteins were dissolved in TRIzol lysates or distilled water containing 10% D_2_O. The pH was adjusted to 2 using HCl, and NH signal assignments from ^1^H-^15^N-labeled HSQC spectra were assigned as described [19].

## Results

### Preparation of nucleic acid-free total cell protein lysates

In order to prepare nucleic acid-free total protein lysates from cultured mammalian cells under native conditions, we removed nucleic acids using three different approaches; selective precipitation with polyethylenimine [20], extensive digestion with nuclease, and chromatographically using an anion-exchange column. Unfortunately, neither method produced a satisfactory yield or purity. In contrast, phenol-chloroform extraction was efficient at ensuring total separation of nucleic acids and denatured total cell proteins. The guanidinium thiocyanate-phenol-chloroform mixture that constitutes TRIzol reagent, that is regularly used for RNA preparation [21], was used to homogenize cells, and proteins extracted using this reagent have been successfully recovered for proteomic research [22]–[24]. In this extraction procedure, proteins are fractionated into the organic phase and precipitated by addition of 2-propanol (Fig. 1), and 90% of total cellular proteins can be recovered, which is considerably higher than was achieved by homogenizing cells directly in 8 M Urea (Fig. 2A). After extensive washes with 0.3 M guanidine hydrochloride (GdnHCl)-95% ethanol, or in ethanol, total cellular proteins were recovered as a tightly packed white pellet following centrifugation, which was used directly or stored at −20°C as a wet pellet to avoid the difficulties associated with resuspending dried pellets in denaturant solutions. When dissolved in 6 M GdnHCl, proteins formed a slightly cloudy solution that clarified following reduction with dithiothreitol (DTT). Proteins were successfully solubilized following dialysis against pure water at acidic pH (Fig. 2 and Table 1) to give a yield of approximately 6 mg/mL from HeLa cells. The pH of the TRIzol lysate was between 5 and 5.8, which was the same as the dialysis solution, confirming dialysis had gone to completion. The electrical conductivity of the TRIzol lysate was less than 20 µS/cm, which was estimated to be less than 1 mM of electrolytes and is probably mostly residual GdnHCl. All Trizol lysates confirmed to show UV absorption spectrum has a peak maximum at approximately 280 nm. The residual nucleic acids in HeLa TRIzol lysate were less than 1 ng/mL in 1 mg/mL of protein by fluorescent nucleic acids detection methods, thus the lysates were virtually nucleic acids free. As shown in Figure 2A, denatured mammalian proteins in nucleic acid-free water showed unexpectedly high solubility compared with the extensive insoluble aggregation observed in denaturant containing nucleic acids (Fig. 1, 2B). Total cellular proteins from another eukaryote (*Saccharomyces cerevisiae*) and two prokaryotes (*Staphylococcus aureus* and *Escherichia coli*) showed reduced solubility (Table 1). However, low molecular weight (<20 kDa) denatured proteins from *E. coli* were soluble in these conditions, whereas most higher molecular weight (>30 kDa) proteins were insoluble (Figure 2C). Recombinant human β -actin is expressed in inclusion bodies in *E. coli*, and is known to be highly insoluble in the denatured form [25]. This protein remained insoluble in the *E. coli* total protein lysate even in nucleic acid-free conditions (Fig. 2C). In contrast, denatured β-actin from HeLa cells showed high solubility in nucleic acid-free conditions (Fig. 2B). The high solubility and resistance to aggregation of mammalian total cellular proteins in nucleic acid-free pure water compared to prokaryotic proteins (Table 1) presumably reflects an evolutionary divergence, which is consistent with the high abundance of IDPs in eukaryotes but not in prokaryotes.

**Figure 1:** Schematic representation of the preparation of total cell protein lysates.

**Figure 2:** Analysis of total cell protein lysates. **A.** SDS-PAGE of total cell proteins lysed with 8 M urea or precipitated from the organic phase of TRIzol homogenates (an equivalent number of HeLa cells were used in each case). Endogenous proteins were also analyzed using western blotting. **B.** SDS-PAGE of total cell protein TRIzol and GdnHCl lysates. Equivalent amounts of protein in soluble fractions (S) and precipitates (P) following centrifugation were loaded. **C.** SDS-PAGE of TRIzol lysates prepared from *E. coli* BL21(DE3) expressing or not expressing human β-actin.

**Table 1:** Solubility of denatured and nucleic acid-free total cell proteins in pure water.

Source	Solubility in TRIzol lysate (%)*
*H. Sapien, M. musculus* (HeLa, Hek293, B16–F10)	95.9±1.7
*S.cerevisiae* (S288C)	59.1±8.4
*S. aureus* (FDA209p)	47.3±0.9
*E.coli* (BL21(DE3))	32.9±3.0

*Initial protein concentrations were adjusted to 1 mg/mL before dialysis.

### Effect of additives on the solubility of TRIzol-solubilized proteins from HeLa cells

Nucleic acids at a concentration of 100−300 µM of phosphate group (30–100 µg/mL) induced precipitation of TRIzol-solubilized proteins from HeLa cells. Interestingly, the triphosphate group of dNTPs appeared to be a strong inducer of precipitation of denatured proteins, whereas monophosphate anions showed no such effect in the concentration range studied (Fig. 3A). The ionic strength was also important for solubility; the solubility of proteins in physiological saline decreased to 30% (Fig. 3B). However, non-ionic solutes such as sugars did not affect protein solubility (Fig. 3C), indicating that coulomb interactions between denatured proteins and additives contributed to protein solubility in TRIzol lysates. Although the pH can be an important factor affecting the net charge of protein molecules, this proved difficult to determine to analyze here, because addition of ionic buffers rapidly induced protein aggregation at all pH values tested.

**Figure 3:** Effect of additives on protein solubility in HeLa cell TRIzol lysates. The solubility of proteins remaining after addition of nucleic acids (**A**), sodium chloride (**B**) or carbohydrates (**C**) was determined.

### Protein conformation in TRIzol lysates

To confirm that proteins were completely denatured in TRIzol lysates, HEK293 cells expressing Luciferase or GFP were examined. As shown in Figure 4, both cell types were successfully lysed in Glo Reporter Lysis Buffer (GLB, Promega) under native conditions in which the reporter protein function was maintained. While ensuring the same number of each cell type was used, reporter proteins were successfully recovered in soluble but denatured (non-functional) form in TRIzol lysates. In a previous study, immunoglobulin light chain derived amyloidogenic 3Hmut at pH 2 [19] and *S*-carboxylmethylated mouse lysozyme at pH 5 [17] were confirmed to be fully disordered using heteronuclear NMR spectroscopy [18], [26]. Using these disordered proteins as probes, ^1^H-^15^N heteronuclear single quantum coherence (HSQC) spectra were compared for HeLa TRIzol lysates. As shown in Figure 5, the overall spectra for both proteins exhibited similar crowded resonances indicative of fully denatured proteins. These results confirmed that the proteins in the HeLa cell lysates were fully unfolded and highly soluble.

**Figure 4:** Biological activity of reporter proteins in physiological buffer or TRIzol lysates. Hek293 cells expressing either GFP or Luc were directly lysed in physiological Glo Lysis buffer (GLB) or TRIzol, and GFP or Luc activity were measured. Reporter proteins were verified by western blotting.

**Figure 5:** Effect of water soluble denatured protein mixtures on the solution structure of intrinsically disordered proteins. ^1^H-^15^N HSQC spectra of the intrinsically disordered 3HmutWil and *S*-carboxymethylated mouse lysozyme in the absence (black) and presence (red) of HeLa cell TRIzol lysates. Assignments of 3HmutWil in the absence of lysate are indicated.

## Discussion

In this study, we observed that fully denatured mammalian total cell protein mixtures showed unusually high solubility in nucleic acid-free pure water. This unusual solubility appeared to be characteristic of higher eukaryotes, since proteins from a lower eukaryote (yeast) and two prokaryotes were largely aggregated under comparable conditions. This observation likely reflects a key evolutionary divide since IUPs are known to be highly abundant in mammalian cells [10], [11]. Within the single-celled organisms studied, denatured proteins from the eukaryote *Saccharomyces cerevisiae* showed higher solubility than did those from two prokaryotes (Table 1). This trend was consistent with previous studies on IDPs from *Saccharomyces cerevisiae* and *E. coli* [27]. Therefore, in a salt-free and nucleic acid-free environment, the solubility of denatured proteins is highly correlated with the flexibility of the polypeptide and the proportion of hydrophilic residues in the protein chain.

Reconstitution of nucleic acids into TRIzol lysates from the HeLa cells indicated that these polyanionic macromolecules strongly promote the aggregation of denatured proteins. As shown in Figure 3A, tRNA, which is a tightly folded molecule, induced protein aggregation to a lesser degree than did dNTPs that have exposed phosphate groups. Thus, the electrostatic interactions between nucleic acids and denatured protein molecules could be a strong trigger for protein aggregation. This may explain why mammalian recombinant proteins frequently aggregate in bacterial cells. In our previous study, recombinant proteins isolated from bacterial inclusion bodies were found to be tightly associated with nucleic acid [15].

The ionic strength of TRIzol lysates also affected protein solubility significantly (Fig. 3B). Unfolded purified proteins, including integral membrane proteins, have been successfully solubilized in pure water previously [6], [7], [28]–[30]. Furthermore, the structural and dynamic properties of proteins in 8 M urea and pure water were shown to be similar using NMR [31]. Soluble proteins in pure water are predicted to be highly flexible due to strong intramolecular and intermolecular electrostatic repulsion [30]. In this study, pure water had a pH of 5.6, presumably due to the atmospheric carbon dioxide concentration. At this pH, ionizable groups on Lys, Arg, His, Asp, and Glu residues are potentially fully charged in the absence of counter ions, which maximizes the hydration of unfolded proteins. The high entropy of the denatured proteins in the HeLa cell TRIzol lysates is presumably the reason for the high solubility. Since aggregation requires productive collisions between protein molecules, enthalpy-entropy compensation theory can explain the unusually high solubility of denatured mammalian proteins in pure water [32], [33].

Although the detailed mechanism is unclear, flexible polypeptide chains classified as IDPs may competitively suppress intermolecular interactions between otherwise insoluble hydrophobic polypeptides. Mammalian proteins in TRIzol lysates retained solubility for more than 6 months at 4°C. Importantly, approximately 30% of fully disordered proteins in mixtures from human cells maintained solubility in physiological saline (Fig. 3B). Competitive suppression of protein aggregation may partially explain the extraordinarily high solubility of mammalian proteins in living cells.

Upon screening of aggregation-prone protein domains, highly charged intrinsically disordered flexible sequences termed entropic bristles served as effective solubilizers in fusion partner proteins [33]–[35]. This suggests that disordered regions in IDPs enhance protein solubility via entropic effects, and pure water may enhance this effect. Chemical protein cationization of Cys residues is a powerful approach for solubilization of denatured proteins [17], [36], [37], which also enhances protein flexibility via electrostatic effects. Enhancing protein flexibility therefore appears to be a productive strategy for increasing the solubility of disordered proteins.

Solubilization of proteins is essential for their use in biotechnological and medical applications. Maintaining the biologically active ‘native’ conformation is the preferred approach for soluble proteins. In the case of denatured proteins, especially those of mammalian origin, nucleic acid-free pure water may be a useful solvent for the alternative approach of solubilizing disordered proteins. This alternative approach could be applied in numerous ways. For example, surgically removed cancer tissues contain immunologically important antigens that induce cancer immunity [38]–[40], and the insoluble fraction of tumor cell homogenates in PBS lysed by sonication contain tumor antigens eliciting cytotoxic T-lymphocytes [41]. The method of extracting denatured proteins in high yield established in this study may therefore be useful for preparation of cancer vaccines.
